# A Novel Identified Peptide Hormone “Metabolitin” Attenuates Lipid Absorption in the Small Intestine of Diabetic Mice with Nonalcoholic Fatty Liver Disease by Regulating Neurotensin and AMPK Signaling Pathway

This article has been retracted.

**DOI:** 10.1155/2021/8386848

**Published:** 2021-09-28

**Authors:** Peng Xu, Shanjuan Wang, Dongyue Pang

**Affiliations:** ^1^Gastroenterology Department, Jiading District Central Hospital Affiliated Shanghai University of Medicine & Health Sciences, Shanghai, China; ^2^Endocrine Department, Jiading Branch of Shanghai General Hospital, Shanghai, China

## Abstract

**Aim:**

The purpose of this study was to explore the effect of a novel identified peptide hormone “metabolitin” on lipid absorption in the small intestine of mice with type 2 diabetes mellitus (T2DM) and nonalcoholic fatty liver disease (NAFLD) and potential mechanisms.

**Methods:**

T2DM was induced in mice by 4–6 weeks of high-fat diets followed by intraperitoneal injection of 35 mg/kg STZ. NAFLD was induced in diabetic mice by a month of high-fat diets. Oral administration of 4 pmol/g or 12 pmol/g metabolitin every two days was performed during one-month high-fat diets. Triglyceride (TG) and total cholesterol (TC) detection and Oil Red O staining were performed to evaluate lipid absorption. The neurotensin (NT) levels in the intestinal tissues and serum were determined by ELISA. Lipogenesis- and lipolysis-related proteins, AMP-activated protein kinase (AMPK), and p-AMPK were examined by Western blot analysis.

**Results:**

It was found that glucose tolerance test (GTT), insulin tolerance test (ITT), TG, and TC indicated lower levels in the serum of NAFLD/T2DM mice receiving 4 pmol/g and 12 pmol/g metabolitin compared to the mice receiving normal saline (*P* < 0.05). No significant difference was noted in the TC level of the feces among mice with different diets (*P* > 0.05), but compared to NAFLD/T2DM mice with normal saline, the mice administrated with 4 pmol/g and 12 pmol/g metabolitin revealed much higher TG levels in the feces (*P* < 0.05). The results of Oil Red O staining revealed that the intestinal epithelial cells of NAFLD/T2DM mice receiving 12 pmol/g metabolitin indicated resistance to lipid absorption and the area of staining was smaller than that of NAFLD/T2DM mice with normal saline (*P* < 0.05). The NAFLD/T2DM mice receiving 4 pmol/g and 12 pmol/g metabolitin showed a higher extent of p-AMPK concomitant with lower levels of NT in the serum and small intestine than the mice with normal saline (*P* < 0.05). Western blot analysis also suggested that NAFLD/T2DM mice receiving 4 pmol/g and 12 pmol/g metabolitin revealed lower expressions in fatty acid synthase (FAS), acetyl-CoA carboxylase (ACC), stearoyl-CoA desaturase-1 (SCD-1), and sterol regulatory element-binding transcription factor-1 (SREBP1) proteins and higher expressions in carnitine palmitoyltransferase 1 (CPT1), peroxisome proliferator-activated receptor alpha (PPAR*α*), and fatty acid translocase (CD36) proteins than NAFLD/T2DM mice with normal saline (*P* < 0.05).

**Conclusion:**

According to the data we observed, oral administration of metabolitin could attenuate lipid absorption in the small intestine of NAFLD/T2DM mice, which may be a novel therapeutic approach for NAFLD/T2DM.

## 1. Introduction

Nonalcoholic fatty liver disease (NAFLD) is a syndrome characterized by excessive fat accumulation in liver cells (hepatic steatosis ≥5%), which is not caused by alcohol and other definite liver damaging factors. Among them, a small proportion of NAFLD patients could be developed to nonalcoholic steatohepatitis (NASH), which was defined as hepatocyte injury and presence of hepatic fibrosis, and more severe patients may develop cirrhosis and hepatocellular carcinoma, leading to liver-related morbidity and mortality [1, 2]. Although the pathogenesis of NAFLD remains unclear, various aspects such as insulin resistance, lipids, immunity, intestinal flora, genetic factors, and lifestyle are contributing to the process of NAFLD [3]. A study based on PubMed and MEDLINE databases (1989–2015) indicated that the worldwide prevalence of NAFLD was about 25.24%; in addition, the prevalence of NAFLD has been increased with age [4]. In clinical, NAFLD patients are more likely to suffer from metabolic syndrome, such as obesity, insulin resistance, type 2 diabetes mellitus (T2DM), dyslipidemia, and hypertension [5, 6]. Among these complications, T2DM seems to be the essential clinical predictor of adverse clinical reactions, such as advanced liver fibrosis and mortality in NAFLD patients [7, 8]. A systematic review and meta-analysis reported that, among T2DM patients, the global prevalence of NAFLD and NASH was 55.5% and 37.3%, respectively, and about 17.0% advanced fibrosis in patients with NAFLD and T2DM [9]. T2DM patients potentially run high risk of afflicting with NAFLD than nondiabetic populations, with the result of developing end-stage liver diseases, including cirrhosis and hepatocellular carcinoma [10], and it was reported that the prevalence of NAFLD in T2DM was 34%–74% [11]. Accumulated evidence has confirmed the correlation between NAFLD and T2DM, which could elaborate lipid metabolism defects and hepatic triacylglycerol (TG) accumulation processed to insulin resistance (IR) and hyperinsulinemia in NAFLD patients or to pancreatic *β*-cell dysfunction in T2DM patients [12, 13]. Thus, clarifying the metabolic pathway of fatty acids in the liver and body is helpful to develop new target drugs for the prevention and treatment of patients with T2DM and NAFLD. In the past, it has been proved that osteocalcin was associated with the regulation of glucose metabolism [14] and the increase of insulin secretion [15]. Meanwhile, it was found that osteocalcin was related to NAFLD development [16]. However, in recent years, no more progress of osteocalcin was observed in metabolism disorders. A newly identified peptide hormone, nominated as metabolitin, was proved to significantly inhibit intestinal fat absorption in NAFLD mice by oral or intraperitoneal administration [17]. Neurotensin (NT), mainly distributed in the special intestinal endocrine cells of the small intestine, promotes the translocation of fatty acids in the mice intestine through fat intake and release [18]. Research has pointed out that NT attenuated the activation of AMP-activated protein kinase (AMPK) and stimulated the absorption of fatty acids in the mouse [19].

However, few studies were conducted on the mechanism of metabolitin on lipid absorption in mouse small intestine. In view of this, this study intended to establish an obese mice model of T2DM combined with NAFLD and analyze the detailed mechanism of metabolitin on lipid absorption in mouse small intestine based on NT-AMPK signaling pathway, in order to provide a scientific basis for the prevention and treatment of mice with T2DM and NAFLD.

## 2. Materials and Methods

### 2.1. Experimental Animals

A total of 38 C57BL/6J male mice (Hunan SJA Laboratory Animal Co., Ltd., SCXK (F) 2020–0009), aged 7 weeks and weighing 19–21 g, were housed for 7 days with humidity of 60–80% at a temperature of 22 ± 2°C, with the freedom to eat and drink, in the condition of light exposure and avoidance alternately for 12 h, respectively. All animal experiments were conducted under the approval of the Ethics Committee of our hospital and in accordance with the Guide for the Care and Use of Laboratory Animal. Extensive efforts were made to ensure minimal suffering of the animals included in the study.

### 2.2. Establishment of T2DM and NAFLD Models

Among 38 mice, 10 mice selected randomly were fed with a normal diet, and the remaining 28 mice have received a high-fat diet containing 45% fat and 10% fructose (Research Diets Inc., US), to establish the T2DM and NAFLD model. After 4–6 weeks of feeding, the physical signs were detected in all mice. During 8 to 12 weeks, glucose tolerance test (GTT) was performed on the mice with a high-fat diet. The evaluation of successful prediabetic model was performed according to the following criteria: (a) impaired glucose tolerance (IGT) was with a slight change in fasting blood glucose (FBG); (b) blood glucose increased significantly at 15–120 min after glucose loading; (c) features of insulin resistance were revealed after the insulin tolerance test (ITT). The area under curve (AUC) during an oral GTT and ITT was used to evaluate the patterns of glucose and insulin resistance changes. After successful establishment of the prediabetic model, water allowing and food forbidding were carried out in all mice for 12 h. Intraperitoneal injection of 35 mg/kg streptozotocin (STZ) (Sigma-Aldrich, US) was applied to 28 mice at one time, and an equal volume of citric acid/sodium citrate buffer was used to the 10 mice. Blood glucose of all mice was detected randomly by the blood samples from the tail, and the T2DM model was established successfully if the random blood glucose level ≥16.7 mmol/L or FBG >11.1 mmol/L, measured by Accu-Chek Perform (Roche, Germany). After continuing feeding for 30 d, 1 mouse with a normal diet and 1 mouse with a high-fat diet were randomly selected to extract the liver tissue for skin biopsy. The hepatocyte fatty degeneration of the mice was revealed under an inverted microscope (Nikon, Japan), suggesting successful establishment of the NAFLD model.

### 2.3. Sample Collection

Among 28 T2DM/NAFLD mice, 9 mice selected randomly were given oral administration of 4 pmol/g metabolitin (metabolitin is a new polypeptide hormone researched by the Shenzhen Institutes of Advanced Technology Chinese Academy of Sciences) and assigned into the named low metabolitin group, and 9 mice were given oral administration of 12 pmol/g metabolitin and assigned into the named high metabolitin group. The remaining 9 T2DM/NAFLD mice received oral administration of normal saline. The oral administration was performed every other day and lasted for 8 weeks. 38 mice in total fasted the day before sample collection, and blood samples were extracted from each mouse. Eventually, all mice were euthanized by exposure to prolonged inhalation anaesthesia to obtain intestinal samples.

### 2.4. TG Measurement in the Feces

After 7 d of adaptive feeding, feces of all mice were collected and measured for 3 consecutive days. The feces samples were dried in a medical oven at 60°C for 24 hours and ground into powder. The solution of chloroform (1 ml) and methanol prepared in the ratio of 2 : 1 was added to 100 mg fecal powder and then centrifugated in the condition of 1 × 10^6^ g to extract the lipid in the lower layer. The TG and total cholesterol (TC) were detected by an automatic biochemical analyzer (Roche, Germany).

### 2.5. Oil Red O Staining

10 min *μ*l/g olive oil was orally taken in after the mice were treated with 12 pmol/g of metabolitin for 30 min, and the mice were euthanized by exposure to prolonged inhalation anaesthesia to get the small intestine after administration in 30 min. The anterior tissue of small intestine was rinsed with precooled phosphate buffer and fixed in 10% formaldehyde. After formaldehyde on the tissue was completely dried, the tissue was fully soaked by optimal cutting temperature compound (OCT) and precooled immediately. Briefly, the slices of tissue with 4–6 *μ*m were placed on siliconized slides, then immersed in 60% isopropanol, and stained with Oil Red O (Sigma-Aldrich, US) for 10 minutes, respectively, followed by differentiation for 3–10 seconds using 60% isopropanol. Finally, the tissue was stained with Mayer's hematoxylin solution for 1 min and sealed with neutral gum. The red area in the tissue was quantified by real-time PCR (Roche, Germany) and analyzed by Image J software.

### 2.6. Neurotensin (NT) Detection

NT detection of the serum and small intestine in the mice was carried out by microplate reader (BIO-RAD, USA) using enzyme-linked immunosorbent assay (ELISA) kits.

### 2.7. Protein Expression Detection by Western Blotting

The small intestine tissue (0.5 g) was homogenized by lysis buffer (700 *μ*L) (Shanghai Yanxi Biotechnology Co., Ltd, CN) in the dry ice for 30 min at 4°C and then centrifuged for 10 min with the speed of 15000 rpm/min to get protein samples. The optical density (OD) value of protein samples and the protein concentration were determined by bicinchoninic acid (BCA) protein assay kits (Shanghai Yanxi Biotechnology Co., Ltd., CN). The protein samples, diluted with sterilized ddH2O, were mixed with 5 × SDS-PAGE sample loading buffer at the ratio of 4 : 1, denatured at 95°C for 10 min, and then cooled in the refrigerator at −20°C for standby. The protein electrophoresis and membrane transfer were processed as follows: protein samples were fixed in the electrophoresis apparatus, with a constant voltage mode of 80 V for working about 30 min. The voltage was switched to 100 V when separation gel appeared in samples. Taking the protein marker as a reference, the electrophoresis apparatus was shut off according to the separation of molecular weight of the protein samples. The PVDF film, which was equivalent to the size of the protein gel, was preimmersed in carbinol for 3 to 5 min. The protein gel and the PVDF film were assembled in a Sandwich manner and transferred for 90 min with a constant voltage mode of 200 mA. After membrane transfer, the membrane was rinsed with PBST solutions for 3 times, blocked in 5% skim milk for 1 h, and incubated with primary antibodies including anti-AMP-activated protein kinase (AMPK) (1 : 1000, ab32047, Abcam, Cambridge, UK), anti-p-AMPK (1 : 1000, ab133448, Abcam), anti-fatty acid synthase (FAS) (1 : 1000, ab133619, Abcam), anti-acetyl-CoA carboxylase (ACC) (1 : 1000, MA5-24700, Thermo Fisher Scientific, USA), anti-stearoyl-CoA desaturase-1 (SCD-1) (1 : 1000, ab236868, Abcam), anti-sterol regulatory element-binding transcription factor-1 (SREBP1) (1 : 2000, ab28481, Abcam), anti-carnitine palmitoyltransferase 1 (CPT1) (1 : 1000, ab189182, Abcam), anti-peroxisome proliferator-activated receptor alpha (PPAR*α*) (1 : 1000, 178860, Abcam), anti-fatty acid translocase (CD36) (1 : 1000, ab133625, Abcam), and anti-*β*-actin (1 : 10000, ab8226, Abcam) at 4°C overnight. The primary antibody was recovered and rinsed with PBST solution 3 times and mixed with the prepared secondary antibody solution (IgG (1 : 5000)) (Abcam, UK). The final solution was cultivated in the room temperature oscillator for 1 h. Developers A and B, made in the ratio of 1 : 1, were dripped into the PVDF film for exposure and development. Strip images detected were switched into gray image, the strips were adjusted to bright color, and the background was changed to dark area. Line drawing and circling were applied to the strips along the edge, the performance was repeated 3 times to get the average number, and the average of the strips was calculated eventually. The above process was analyzed by Image J software.

### 2.8. Statistical Analysis

SPSS 22.0 and GraphPad Prism 5.0 software were used to analyze the data. The measurement data were expressed as mean ± standard deviation. One-way ANOVA was carried out to compare the data among the groups. *P* < 0.05 indicated that the difference was statistically significant.

## 3. Results

### 3.1. Oral Administration of Metabolitin Attenuated Abnormal Glycolipid Metabolism in T2DM/NAFLD Mice

The serum levels of TC and TG as well as the area under curve (AUC) of GTT and ITT were examined in all mice in order to confirm whether the oral administration of metabolitin can regulate glycolipid metabolism in T2DM/NAFLD mice. As presented in Figures 1(a)–1(e), the mice with oral administration of 4 pmol/g and 12 pmol/g metabolitin were lighter than the T2DM/NAFLD mice; the AUC of GTT and ITT was smaller and TC and TG concentrations were lower in the mice with oral administration of 4 pmol/g and 12 pmol/g metabolitin than those in the T2DM/NAFLD mice (*P* < 0.05), suggesting that oral administration of metabolitin prevented abnormal glycolipid metabolism in T2DM/NAFLD mice.

### 3.2. Oral Administration of Metabolitin Inhibited Intestinal Absorption of Fatty Acids in T2DM/NAFLD Mice

Further studies, involving the TG and TC value in the feces of mice, and determination of Oil Red O staining were processed to analyze the intestinal absorption of fatty acids in the mice. It was found that the TG level in the feces of the mice receiving 4 pmol/g and 12 pmol/g metabolitin was obviously higher than that in the model mice (*P* < 0.05, Figure 2), and the TC level in the feces was manifested a slight difference in the mice treated with normal diet and high-fat diet (*P* > 0.05), which indicated that the metabolitin inhibited the TG absorption in the mice. According to the result of the determination of Oil Red O staining, the mice treated with normal saline plus normal saline revealed the fat ratio of 0.02 ± 0.01, the mice receiving normal saline plus Oil Red O indicated the fat ratio of 10.26 ± 1.03, and the mice receiving 12 pmol/g metabolitin plus Oil Red O showed the fat ratio of 2.18 ± 0.07. It was suggested that the absorption of fatty acids in the intestinal epithelial cells of the mice was inhibited by the oral administration of metabolitin.

### 3.3. Oral Administration of Metabolitin Activated the NT-AMPK Signaling Pathway in T2DM/NAFLD Mice

AMPK, as one of the most important molecular energy sensors in eukaryotic cells, plays a leading role in regulating cellular energy balance, and the activity of AMPK is associated with controlling a variety of metabolic processes and liking cell metabolism with energy utilization. NT is an endogenous tridecapeptide, expressed in the central and peripheral nervous system. It is involved in appetite, memory, and physiological activities, as well as lipid metabolism. We detected the protein expression of the mice by Western blot analysis, and as listed in Figures 3(a)-3(b), it was observed that the level of p-AMPK in the mice receiving 4 pmol/g and 12 pmol/g metabolitin was significantly higher than that in the model mice (*P* < 0.05). On the basis of the results of ELISA, compared to the model mice, we found that the NT level of the serum and small intestine revealed a significant decrease in mice receiving oral administration of 4 pmol/g and 12 pmol/g metabolitin (Figures 3(c)–3(e)). These data suggested that oral administration of metabolitin activated the NT-AMPK signaling pathway in T2DM/NAFLD mice.

### 3.4. Oral Administration of Metabolitin Affected Expressions of Lipogenesis- and Lipolysis-Related Proteins in T2DM/NAFLD Mice

Lipid tissue is crucial for metabolic homeostasis, which regulates lipid storage and mobilization on different condition of nutrition. It is associated with insulin coordination and triggered kinase signal cascade to regulate various metabolic proteins, resulting in anabolic processes such as lipogenesis and lipolysis. In this study, compared to the model mice, Western blot analysis suggested that the mice with oral administration of 4 pmol/g and 12 pmol/g metabolitin revealed obviously lower expressions in lipogenesis-related proteins including FAS, ACC, SCD-1, and SREBP1, compared with the model mice (*P* < 0.05, Figure 4). In addition, it was found that lipolysis-related proteins including CPT1, PPAR*α*, and CD36 manifested significantly higher expressions in the mice receiving 4 pmol/g and 12 pmol/g metabolitin compared with the model mice (*P* < 0.05, Figure 5). These data uncovered that oral administration of metabolitin affected expressions of lipogenesis- and lipolysis-related proteins in T2DM/NAFLD mice.

## 4. Discussion

NAFLD is a common liver disease excluding excessive drinking and other clear liver damaging factors. It has a wide spectrum that ranges from simple fatty liver to NASH, cirrhosis, and hepatocellular carcinoma [20]. NAFLD is a multisystem disease that affects many extrahepatic organ systems and interacts with the regulation of multiple metabolic pathways. The prevalence of liver-related morbidity and mortality is related to NAFLD, with the result of increasing risks of other chronic diseases, such as T2DM and cardiovascular disease [4]. A large amount of epidemiological and experimental evidence has suggested that IR is involved in the occurrence of NAFLD and T2DM [21]. Of course, further research is needed to deeply understand the pathophysiological correlation between NAFLD and T2DM. Despite many attempts, the potential molecular mechanism leading to NAFLD and T2DM is still largely unknown. In the present study, we aimed to establish a mice model with NAFLD and T2DM and further explore the mechanism of a new protein hormone named metabolitin in the mice according to the NT-AMPK signaling pathway.

Due to metabolic disorders such as obesity and T2DM, organic factors secreted by adipose tissue and liver may affect the occurrence and development of NAFLD. Lipid accumulation in hepatocyte plays an important role in the pathogenesis of NAFLD [22]. There are two main sources of fatty acids in the liver. One comes from intestinal absorption or the free fatty acids decomposed by TG in adipose tissue, which are transported to the liver through blood. The other originated from the process of excess carbohydrates converted by hepatocytes [23].

In this study, the serum levels of TC and TG, as well as the AUC of GTT and ITT, were significantly declined in the mice with oral administration of 4 pmol/g and 12 pmol/g metabolitin. It suggested that oral administration of metabolitin could be associated with regulation of glycolipid metabolism in the mice, and the outcomes may be related to glucagon-like peptide-1 (GLP-1) secretion promoted by metabolitin. GLP-1 is a hormone mainly produced by intestinal L cells and belongs to incretin. GLP-1 has been well established in reducing body weight and lowering blood sugar through inhibiting gastrointestinal peristalsis and gastric juice secretion and enhancing insulin secretion [24]. A variety of studies have confirmed that impaired glucose homeostasis was reflected by higher AUC of GTT and ITT [25, 26]. Furthermore, the concentration of TG and TC in the feces of all mice was detected to confirm the regulation of metabolitin on lipid metabolism. It was found that, compared to the mice with normal saline, the mice treated with 4 pmol/g and 12 pmol/g metabolitin revealed a significant increase in the level of TG and a slight change in the TC level, indicating that metabolitin can significantly inhibit intestinal absorption of TG rather than TC. TG is the main form of storage and transport of fatty acids in cells and plasma, which occurs mainly in hepatocytes [27]. Under normal conditions, the liver only stores a small amount of TG. However, in the case of obesity and NAFLD, the metabolism disorder of fatty acid in the liver occurs, resulting in excessive accumulation of TG in hepatocytes [28]. In the study of obese mice, the accumulations of TG and TC have been proven to be associated with steatosis and NAFLD as indicated by Lee et al. [29]. The digestion and absorption of lipids are mainly associated with the small intestine, especially in the proximal small intestine. Additionally, some aspects, including dietary options, intestinal endocrine response, choleresis, pancreatic hormone secretion, and intestinal cells, contributed to absorption of lipids and other dietary nutrients [30].

This study designed an acute intestinal experiment. The proximal small intestine of the mice with 12 pmol/g metabolitin was detected by Oil Red O staining. The outcomes revealed that the mice were resistant to lipid absorption, and the area of staining was significantly smaller than the mice with normal saline. It indicated that acute stimulation of metabolitin was a great contributor to inhibition of fatty acid. Oil Red O staining is a gold standard for quantifying steatosis in the liver, which has been confirmed in a variety of studies [31, 32].

Intestinal hormones are an essential part of regulating intestinal lipid absorption. NT is a 13 amino acid polypeptide mainly located in enteroendocrine cells of the small intestine and released by fat intake. Li J. et al. have pointed out that NT-deficiency mice revealed a significant reduction in intestinal fat absorption; additionally, NT directly inhibits the AMPK signaling pathway of epithelial cells, leading to promoting the absorption of fatty acids in intestinal cells [19]. The outcomes were similar to ours, suggesting that the content of p-AMPK was significantly higher, and the NT level of serum and small intestine was reduced obviously in the mice with 4 pmol/g metabolitin and 12 pmol/g metabolitin. These data demonstrated that metabolitin may inhibit the process of intestinal lipid absorption by promoting the activation of AMPK and reducing NT release. Teng et al. [17] also reported that metabolitin can control NT secretion through the AMPK signaling pathway to inhibit TG absorption in intestine, which might be a potential candidate for the treatment of NAFLD.

FAS, ACC, SCD-1, and SREBP1 are important transcription factors regulating fatty acid synthesis. CPT1, PPAR*α*, and CD36 are associated with regulating the oxidation, transport, and uptake of fatty acids *β* [33]. Further analysis in this study showed that the protein expression of SREBP1 and its downstream proteins involving FAS, ACC, and SCD-1 in the mice were downregulated markedly after oral administration of 4 pmol/g and 12 pmol/g metabolitin, which was supported by another study, suggesting that expression increase of FAS, ACC, SCD-1, and SREBP1 was inhibited by diosgenin, so as to ameliorate gestational diabetes [34]. Additionally, we observed that the expression of PPAR*α*, CPT1, and CD36 was significantly upregulated in the mice treated with metabolitin. The findings were close to previous studies. Zhang et al. [35] revealed that IR improvements were related to the increased activity of PPAR*α*, CPT1, and CD36 protein. The research on obese mice has proved similar outcomes as well [36]. All these outcomes from others indirectly confirmed that oral administration metabolitin contributed to biological regulation. Briefly, metabolitin can inhibit intestinal lipid absorption by regulating intestinal hormones and indirectly attenuate intestinal lipid absorption by reducing lipid deposition.

In summary, metabolitin regulates the protein expressions of lipid metabolism through activating the NT-AMPK signaling pathway, leading to lightening lipid accumulation and reducing the absorption of fatty acids (Figure 6), which provides more possibilities for the research and development of new drugs for T2DM combined with NAFLD.

## Figures and Tables

**Figure 1:** Oral administration of metabolitin attenuated abnormal glycolipid metabolism in T2DM/NAFLD mice. (a) The mouse weight at indicated time points (0–12 weeks). (b) The AUC during the oral GTT. (c) The AUC during the oral ITT. (d) The concentration of TC in the mouse serum. (e) The concentration of TG in the mouse serum. ^*∗∗*^*P* < 0.01 compared to the normal group; ^##^*P* < 0.01 compared to the model group.

**Figure 2:** Oral administration of metabolitin increased the level of TG in the feces of T2DM/NAFLD mice. ^*∗∗*^*P* < 0.01 compared to the normal group; ^##^*P* < 0.01 compared to the model group.

**Figure 3:** Oral administration of metabolitin activated the NT-AMPK signaling pathway in T2DM/NAFLD mice. (a, b) The p-AMPK/AMPK in the mouse intestinal tissues was evaluated by Western blot analysis. (c, d) The NT level in the serum and feces of the mice after Oil Red O treatment. (e) The NT level in the serum of the mice after oral administration of metabolitin. In (b) and (e), ^*∗∗*^*P* < 0.01 compared to the normal group; ^#^*P* < 0.05 and ^##^*P* < 0.01 compared to the model group. In (c) and (d), ^*∗∗*^*P* < 0.01 compared to the saline + saline group and ^##^*P* < 0.01 compared to the saline + Oil Red O group.

**Figure 4:** Oral administration of metabolitin caused reduced expressions of lipogenesis-related proteins including FAS, ACC, SCD-1, and SREBP1 proteins. ^*∗*^*P* < 0.01 compared to the normal group; ^#^*P* < 0.01 compared to the model group.

**Figure 5:** Oral administration of metabolitin caused increased expressions of lipolysis-related proteins including CPT1, PPAR*α*, and CD36 proteins. ^*∗*^*P* < 0.01 compared to the normal group; ^#^*P* < 0.01 compared to the model group.

**Figure 6:** Metabolitin regulates the protein expressions of lipid metabolism through activating the NT-AMPK signaling pathway.

## Data Availability

The data used to support the findings of this study are included within the article.
